RETRACTED

# Establishment of Multiple Parameter Reference Intervals for Different Age Groups in Qingdao, China

**DOI:** 10.1155/2022/1966798

**Published:** 2022-03-09

**Authors:** Huan Wang, Jing Li, Rongrong Dong, Yan Wang, Lixia Chen, Qing Wang

**Affiliations:** ^1^Department of Clinical Laboratory, The Affiliated Hospital of Qingdao University, Qingdao, China; ^2^Clinical Laboratory, Qingdao Women and Children's Hospital Affiliated Qingdao University, Qingdao, China; ^3^Health Management Center, The Affiliated Hospital of Qingdao University, Qingdao, China

## Abstract

In this article, we have explored the establishment of multiple parameter reference intervals for different age groups in Qingdao, China. According to the age of subjects, the healthy adult population of different ages in Qingdao was randomly selected as the research object. According to the age of subjects, they were divided into 18–24-year-old, 25–39-year-old, 40–49-year-old, 50–64-year-old, and >65-year-old groups, respectively. The sample size of each age group was 120 male and female samples, and 60 male and female samples of >65-year-old subjects were selected. The data of subjects were collected, a questionnaire survey was completed, serum samples were collected, and the parameters of male and female groups of different ages in Qingdao were compared. The parameters of the male and female groups were compared in the same age group. The reference intervals of parameters of the male and female groups were compared in different ages. There were significant differences in the levels of FBG, AST, BUN, Cr, Hb, FT3, TT3, FT4, TT4, VB12, PROG, CYFRA 21-1, and SCC among men of different ages (*P* < 0.05). Among them, the levels of FBG, AST, BUN, VB12, CYFRA 21-1, and SCC in >65-year-old men were significantly higher than those in 18–24-years-old men, and the levels of Hb, FT3, TT3, FT4, TT4 in >65-year-old men were significantly lower than those in 18–24-year-old men (*P* < 0.05). There were significant differences in FBG, ALT, AST, BUN, Cr, Hb, TSH, FT3, TT3, FT4, TT4, VB12, CYFRA 21-1, anti-TPO, and ferritin levels among women of different ages (*P* < 0.05). Among them, the levels of FBG, ALT, AST, BUN, and ferritin in women aged >65 were significantly higher than those in women aged 18–24 (*P* < 0.05). The levels of FBG, ALT, AST, BUN, Cr, Hb, FT3, TT3, FT4, TT4, and VB12 in women aged 50–64 were significantly higher than those in women aged 25–39, and the levels of TSH were significantly lower than those in women aged 25–39 and significantly higher than those of the female population aged 40–49 (*P* < 0.05). The levels of ALT, AST, BUN, Cr, Hb, FT3, TT3, FT4 and ferritin in males aged 18–24 were significantly higher than those in females, while the levels of TSH, VB12 in males aged 18–24 were significantly lower than those in females (*P* < 0.05). The levels of FBG, ALT, AST, BUN, Cr, Hb, FT3, TT3, FT4 and ferritin in males aged 25–39 were significantly higher than those in females, while the levels of TSH, VB12, CYFRA 21-1 in males aged 25–39 were significantly lower than those in females (*P* < 0.05). The levels of FBG, ALT, AST, BUN, Cr, Hb, FT3, TT3, FT4, CYFRA 21-1 and ferritin in males aged 40-49 were significantly higher than those in females, and the levels of VB12, anti-TG, anti-TPO in males aged 40-49 were significantly lower than those in females (*P* < 0.05). The levels of FBG, ALT, BUN, Cr, FT3, TT3 and ferritin in males aged 50-64 were significantly higher than those in females, while the levels of VB12, anti-TG in males aged 50-64 were significantly lower than those in females (*P* < 0.05). The levels of Cr, Hb and ferritin in males >65 years old were significantly higher than those in females (*P* < 0.05). The reference intervals of various parameters are different among different ages and genders. The establishment of multiparameter reference intervals for different age groups in Qingdao, China, is of great significance for the early diagnosis and evaluation of various diseases in Qingdao, China, so as to reduce the missed diagnosis rate of diseases and improve people's quality of life.

RETRACTED

## 1. Introduction

With the progress of social science and technology, people's lifestyle gradually changes and the incidence of various diseases is rising, seriously affecting people's quality of life and even health. Therefore, early diagnosis, timely detection, and treatment are of great significance to improve the quality of life of patients and patient prognosis. The reference interval is the value between the upper and lower reference limits, and it is also the most commonly used and reliable decision-making tool in clinics [1]. The correct reference interval plays an important role in the diagnosis of disease and health assessment [2]. In the world, due to geographical differences and ethnic and environmental differences, the reference ranges of various indicators of the Chinese population are different from those in western countries; however, the systematic research level of the reference interval of the routine clinical laboratory test items in China is relatively backward, so it is important to establish the reference interval suitable for the population location in China to find and treat the disease in time [3]. Qingdao is located in the north of China, near the sea, and has its unique eating habits.

Currently, the World Health Organization (WHO) defines health as a state of good health that includes physical, mental, and social aspects [4]. People's immune function gradually decreases with age, which increases the risk of diseases, especially chronic diseases [5]. However, the reference range is sensitive to many factors, such as region, environment, economic level, living habits, age, and sex [6]. Therefore, it is of great significance to establish an accurate, applicable, and reliable reference range for the local population to judge the patient's diseases and treat them in time.

RETRACTED

In this paper, we have explored the establishment of multiple parameter reference intervals for different age groups in Qingdao, China. For this purpose, according to the age of subjects, a healthy adult population of different ages in Qingdao was randomly selected as the research object. According to the age of subjects, they were divided into 18–24-year-old, 25–39-year-old, 40–49-year-old, 50–64-year-old, and >65-year-old groups, respectively. The sample size of each age group was 120 male and female samples, and 60 male and female >65-year-old subjects were selected. The data of subjects were collected, a questionnaire survey was completed, serum samples were collected, and the parameters of male and female groups of different ages in Qingdao were compared.

The rest of this article are arranged as follows.

In Section 2, the proposed methodology, i.e., multiple parameter reference intervals for different age groups in Qingdao, China, is described in detail along with a detailed discussion of the possible selection and rejection criteria for the patients of different ages. Experimental results of the proposed approach are presented in Section 3, followed by a detailed discussion section. Finally, concluding remarks and possible future directives are provided in the last section. Lastly, the references used in this article are presented.

## 2. Materials and Methods

### 2.1. Patients or Subjects

The subjects were randomly divided into five groups: 18–24-year-old group, 25–39-year-old group, 40–49-year-old group, 50–64-year-old group, and >65-year-old group; the sample size was 120 males and 120 females of each age group and 60 males and 60 females of >65-year-old group.

### 2.2. Grouping Criteria

- Fasting for at least 10 hours before blood collection
- Age ≥18 years old, male and female
- No history of cardiovascular, liver, kidney, respiratory, blood and lymph, endocrine, immune, mental, nervous, gastrointestinal system, and other chronic or serious diseases
- Voluntarily signing the informed consent form before the test and having a good understanding of the content, procedure, and possible adverse reactions of the test
- This study is in line with the medical ethics principles.

RETRACTED

### 2.3. Exclusion Criteria

- People with diabetes who are on oral medication or insulin
- Patients with chronic liver and kidney disease who are abnormal or/and have a history of complaints
- Abnormal blood pressure (≥140/90 mmHg)
- Hospitalized or operated on in the last 4 weeks
- Donated more than 200 ml of blood in the first three months
- Nearly 2 weeks of taking oral contraceptives, hormones, drugs
- A pregnant woman who has given birth during lactation or in the previous year
- Participating in other clinical trials of the same researcher in the last 12 weeks
- Three days of vigorous exercise before blood collection (such as running a marathon and strenuous gym exercise)
- The researchers concluded that participation in the study may have led to illness or discomfort or other illnesses or conditions that may affect the results of the study, such as alcoholism, smoking, obesity, fatigue, or specific occupations.

### 2.4. Research Methodology

Gather information about the subject: gather the information that may be relevant to the subject's health, including demographics information, such as age, sex, marital status, and ethnicity; vital signs such as blood pressure, heart rate, and body temperature; general laboratory examination (such as liver and kidney function and blood sugar); other clinical results.

Fill in the questionnaire, including the history of the disease, recent history of medication, history of surgery, history of allergies, genetic history, blood donation in the last three months, the history of clinical trials, animal breeding, whether oral contraceptives, hormones, menstrual cycle, smoking habits, drinking, and exercise and fitness frequency and intensity.

Blood samples were collected: blood samples were taken from the subjects, at least 2 ml of venous blood from 7 to 10 am on an empty stomach, and the names and batch numbers of the blood vessels and blood needles were recorded to minimize bias in the results. The serum samples were stored in 2 tubes of 1 ml each. The isolation, separation, and cryopreservation of the serum samples should be completed as soon as possible after blood collection.

Fasting blood glucose (FBG), aspartate transaminase (AST), alanine transaminase (ALT), blood urea nitrogen (BUN), creatinine(Cr), hemoglobin(Hb) and other indicators were measured by Hitachi automatic biochemical analyzer. Use the ARCHITECT reagent for cytokeratin fragment 21–1 (CYFRA 21-1), squamous cell carcinoma (SCC), thyroglobulin antibody (anti-TG), thyroid peroxidase antibody (anti-TPO), thyroid-stimulating hormone (TSH), free triiodothyronine (FT3), total triiodothyronine (TT3), free thyroxine (FT4), total thyroxine (TT4), ferritin, vitamin B12 (VB12), male progesterone (PROG) in Abbott's ARCHITECT 2000 platform for centralized detection.

RETRACTED

### 2.5. Observation Index

- The parameters of the male population and female population in different age groups in Qingdao were compared.
- The parameters of the male and female population in the same age group were compared.
- The parameters of reference ranges of the male and female population in different age groups were compared.

### 2.6. Statistical Methods

In this study, we have reviewed the collected data to eliminate possible errors and outliers (using Dixon's test to identify and eliminate *d*/*r* > = 1/3 samples) and added at least 120 samples per analysis group (at least 60 samples over 65 years of age), The results of the experiment can be tested by SPSS Statistical Software. The results conform to the normal distribution. The reference interval can be determined using the normal distribution method (*μ* ± 1.96 s; *μ* is the mean and *S* is the standard deviation) and the percentile method (the reference range is set by selecting the 95% confidence interval, i.e., 2.5th as the lower limit and 97.5 th as the upper limit). The differences in test results among different sex and/or age groups can be analyzed by item.

## 3. Experimental Results and Observations

### 3.1. Comparison of the Related Parameters among Different Age Groups of Males in Qingdao, China

The levels of FBG, AST, BUN, Cr, Hb, FT3, TT3, FT4, TT4, VB12, PROG, CYFRA 21-1, and SCC in different age groups were significantly different (*P* < 0.05), but the levels of ALT, TSH, anti-TG, anti-TPO, and ferritin were not significantly different (*P* > 0.05) The levels of FBG, AST, BUN, VB12, CYFRA 21-1, and SCC in the male population >65 years old were significantly higher than those in the male population 18–24 years old, and the levels of Hb, FT3, TT3, FT4, TT4 were significantly lower than those in the male population 18–24 years old (*P* < 0.05). See Table 1.

### 3.2. A Comparative Study on the Related Parameters among Different Age Groups of Women in Qingdao, China

The levels of FBG, ALT, AST, BUN, Cr, Hb, TSH, FT3, TT3, FT4, TT4, VB12, CYFRA 21-1, anti-TPO, and ferritin in different age groups were significantly different (*P* < 0.05), but the levels of SCC and anti-TG were not significantly different (*P* > 0.05). Among them, the levels of FBG, ALT, AST, BUN, and ferritin in the female population >65 years old were significantly higher than those in the female population 18–24 years old (*P* < 0.05). The levels of FBG, ALT, AST, BUN, Cr, Hb, FT3, TT3, FT4, TT4, and VB12 in the 50–64-year-old females were higher than those in the 25–39-year-old females, and the levels of TSH were lower than those in the 25–39-year-old females and higher than those in the 40–49-year-old females (*P* < 0.05). See Table 2.

RETRACTED

### 3.3. A Comparative Study of Correlation Parameters between Males and Females in the Same Age Group of 18–24 Years

The levels of ALT, AST, BUN, Cr, Hb, FT3, TT3, ferritin, and FT4 in males aged 18–24 were significantly higher than those in females, and the levels of TSH, VB12 were significantly lower than those in females (*P* < 0.05). There were no significant differences in the levels of FBG, TT4, CYFRA 21-1, SCC, anti-TG, and anti-TPO between the two sexes (*P* > 0.05). See Table 3.

### 3.4. A Comparative Study of Correlation Parameters between Male and Female in the Same Age Group of 25–39 Years Old

The levels of FBG, ALT, AST, BUN, Cr, Hb, FT3, TT3, ferritin and FT4 in males aged 25–39 were significantly higher than those in females, and the levels of TSH, VB12, CYFRA 21-1 were significantly lower than those in females (*P* < 0.05). There was no significant difference in the levels of TT4, SCC, anti-TG, and anti-TPO between the sexes (*P* > 0.05). See Table 4.

### 3.5. Comparison of Correlation Parameters between 40–49-Year-Old Men and Women

The levels of FBG, ALT, AST, BUN, Cr, Hb, FT3, TT3, FT4, ferritin and CYFRA 21-1 in males aged 40-49 were significantly higher than those in females, and the levels of VB12, anti-TG, anti-TPO were significantly lower than those in females (*P* < 0.05). There was no significant difference in the TSH, TT4, and SCC levels between the sexes (*P* > 0.05). See Table 5.

### 3.6. A Comparative Study of Correlation Parameters between Male and Female in the Same Age Group of 50–64 Years Old

The levels of FBG, ALT, BUN, Cr, FT3, TT3 and ferritin in males aged 50–64 were significantly higher than those in females, and the levels of VB12, anti-TG were significantly lower than those in females (*P* < 0.05). There were no significant differences in AST, TSH, FT4, TT4, CYFRA 21-1, SCC, and anti-TPO levels between the two sexes (*P* > 0.05). See Table 6.

### 3.7. Correlation Parameter Comparison between Male and Female in the Same Age Group of > 65 Years Old

The levels of Cr, Hb and ferritin in males >65 years old were significantly higher than those in females (*P* < 0.05). There were no significant differences in the levels of FBG, ALT, AST, BUN, TSH, FT3, TT3, FT4, TT4, CYFRA 21-1, SCC, anti-TG, and anti-TPO between the sexes (*P* > 0.05). See Table 7.

### 3.8. The Reference Range of Male Parameters in Different Age Groups

The reference intervals of parameters for different age groups were different. The reference intervals of FBG, AST, ALT, BUN, Cr, Hb, TSH, FT3, TT3, FT4, TT4, VB12, PROG, CYFRA 21-1, SCC, anti-TG, anti-TPO, and ferritin are shown in Table 8.

RETRACTED

### 3.9. Reference Range of Parameters for Different Age Groups of Women

The reference ranges of parameters for different age groups were different. The reference ranges of FBG, AST, ALT, BUN, Cr, Hb, TSH, FT3, TT3, FT4, TT4, VB12, PROG, CYFRA 21-1, SCC, Anti-Tg, Anti-TPO, Ferritin were shown in Table 9.

## 4. Discussion

Currently, WHO defines health as a state of good health that includes physical, mental, and social aspects [4]. People's immune function gradually decreases with age, which increases the risk of diseases, especially chronic diseases. Reference interval refers to the interval between the lower and upper reference limits. It is an important tool for diagnosis, treatment, prognosis, disease prevention, and health detection. It is also the most widely used medical decision tool in clinics [5]. However, the reference range is sensitive to many factors, such as region, environment, economic level, living habits, age, and sex [6]. Therefore, it is of great significance to establish an accurate, applicable, and reliable reference range for the local population to judge the patient's diseases and treat them in time.

In this study, 1080 adults aged 18 and over in Qingdao, China, were randomly selected to estimate the reference limit of 90% confidence interval using the nonparametric method and divided into five age groups according to age: 18–24 years, 25–39 years, 40–49 years, 50–64 years and >65 years, ensuring that each age group has the same number of participants, with a sample size of at least 120 males and 120 females per age group and a sample of at least 60 men and 60 women over 65 years of age that met the criteria set by the Clinical and Laboratory Standards Institute(CLSI). Because the indexes of FBG, AST, ALT, BUN, Cr, Hb, TSH, FT3, TT3, FT4, TT4, VB12, PROG, CYFRA 21-1, SCC, anti-TG, anti-TPO, and ferritin are of great significance in clinical work to provide a reference for clinical accurate diagnosis and treatment, in this study, the above-mentioned index is taken as the research index.

With the change in people's lifestyles, the incidence of diabetes gradually increases and tends to be prevalent in younger populations. FBG was used as an index to detect fasting blood glucose, and the abnormal level of FBG was significantly correlated with abnormal glucose regulation [7]. Some studies have shown that the increase of FBG levels is an important stage that directly or indirectly leads to the occurrence and death of cardiovascular events [8]. AST, ALT, BUN, Cr, and so on are among the most commonly used indexes for detecting liver and renal function in clinics [9, 10]. The levels of AST, ALT, BUN, and Cr increased obviously when the liver and kidney were damaged. Cr is a product of muscle metabolism [11]. Under normal circumstances, the amount of Cr produced in the body is relatively constant, but when the kidney function is seriously damaged, the level of Cr rises obviously. The results showed that the levels of AST, ALT, BUN, and Cr were significantly different in different sex and age groups. The ALT reference level in Qingdao was significantly higher than that in Haikou [12]. This may be due to more alcohol intake, heavier diet, a faster pace of life, and greater work stress in Qingdao, resulting in a higher ALT reference range in the region.

RETRACTED

Thyroid disease is an endocrine system disease with a statistically higher probability of thyroid disease worldwide; the study found [13] that there were significant differences in FT3, TT3, FT4, and TT4 between the ages of 18–24, 25–39, 40–49, and 50–64, but there was no significant difference in the age of >65. Therefore, it is significant to set the reference interval by age group.

With the trend of changing lifestyles and population aging, the morbidity and mortality rates of malignant tumors are increasing year by year, which has become a serious disease affecting people's life and health. Therefore, the early diagnosis and treatment of tumors can improve the therapeutic effect, prolong the survival time, and improve the prognosis. Tumor markers can rapidly and effectively diagnose the early tumor and provide important evidence for early treatment of tumor [14]. Ideal serum tumor markers should have high sensitivity and specificity. It was found that [15] the concentrations of CYFRA 21-1, SCC, and ferritin were low under normal conditions, but the levels of CYFRA 21-1, SCC, and ferritin increased significantly when the cells became cancerous. This study found that the CYFRA 21-1 levels increased significantly with age. The SCC levels were the highest in males aged over 65 and highest in females aged 18-39. There were significant differences in ferritin levels between the sexes in different age groups. Therefore, it is very important to establish the reference intervals of CYFRA 21-1, SCC, and ferritin for the early diagnosis of tumor.

In conclusion, the establishment of multiparameter reference ranges for different age groups in Qingdao, China, is of great significance for the early diagnosis and evaluation of various diseases in Qingdao, China, to reduce the rate of missed diagnosis and improve people's quality of life.

## 5. Conclusion and Future Work

In this study, 1080 adults aged 18 and over in Qingdao, China, were randomly selected to estimate the reference intervals by the nonparametric method and divided into five age groups according to age: 18–24 years, 25–39 years, 40–49 years, 50–64 years and >65 years, ensuring that each age group has the same number of participants, with a sample size of at least 120 males and 120 females per age group and a sample of at least 60 men and 60 women over 65 years of age that met the criteria set by the CLSI. Because the indexes of FBG, AST, ALT, BUN, Cr, Hb, TSH, FT3, TT3, FT4, TT4, VB12, PROG, CYFRA 21-1, SCC, anti-TG, anti-TPO, and ferritin are of great significance in clinical work, to provide a reference for clinical accurate diagnosis and treatment, in this study, the above-mentioned index is taken as the research index. The establishment of multiparameter reference ranges for different age groups in Qingdao, China, is of great significance for the early diagnosis and evaluation of various diseases in Qingdao, China, to reduce the rate of missed diagnosis and to improve people's quality of life.

RETRACTED

In the future, we are eager to extend the operational capacity of the proposed study to other diseases or different groups.

## Figures and Tables

**Table 1:** Comparison of the related parameters among different age groups of males in Qingdao, China ($\bar{x}$ ± *s*).

Groups	18–24 (*n* = 120)	25–39 (*n* = 120)	40–49 (*n* = 120)	50–64 (*n* = 120)	>65 (*n* = 60)	*F*	*P*
FBG (mmol/L)	4.71 ± 0.35	4.66 ± 0.42	4.95 ± 0.46^ab^	5.18 ± 0.55^abc^	5.31 ± 0.78^abc^	37.304	<0.001
ALT (IU/L)	20.76 ± 12.63	23.56 ± 20.76^a^	22.26 ± 20.76	21.24 ± 9.58	19.34 ± 11.24^b^	2.203	0.067
AST (IU/L)	17.85 ± 4.88	19.03 ± 6.12	18.90 ± 5.35	19.26 ± 4.91^a^	20.95 ± 6.32^abcd^	3.778	0.005
BUN (mmol/L)	5.00 ± 0.97	5.15 ± 1.08	5.26 ± 1.09^a^	5.53 ± 1.22^abc^	6.04 ± 1.55^abcd^	11.207	<0.001
Cr (Umol/L)	103.73 ± 7.82	101.35 ± 8.63^a^	100.67 ± 10.06^a^	101.24 ± 9.96^a^	100.88 ± 11.54^a^	2.404	0.049
Hb (g/L)	159.58 ± 8.28	155.60 ± 9.29^a^	156.06 ± 8.27^a^	154.92 ± 9.48^a^	150.08 ± 10.30^abcd^	13.324	<0.001
TSH (uIU/mL)	1.89 ± 1.00	1.78 ± 0.81	1.79 ± 1.29	1.89 ± 1.22	2.18 ± 1.26^bc^	1.763	0.135
FT3 (pmol/L)	4.99 ± 0.46	4.69 ± 0.44^a^	4.63 ± 0.41^a^	4.70 ± 0.42^a^	4.40 ± 0.39^abcd^	24.975	<0.001
TT3 (ng/mL)	1.19 ± 0.14	1.12 ± 0.15^a^	1.09 ± 0.15^a^	1.13 ± 0.16^ac^	1.07 ± 0.16^ad^	12.026	<0.001
FT4 (pmol/L)	14.35 ± 1.27	14.01 ± 1.27^a^	13.78 ± 1.15^a^	13.36 ± 1.24^abc^	13.28 ± 1.13^abc^	15.950	<0.001
TT4 (*μ*g/dL)	8.20 ± 1.11	7.86 ± 1.24^a^	7.71 ± 1.25^a^	7.84 ± 1.26^a^	7.59 ± 1.20^a^	4.081	0.003
PROG (nmol/L)	0.73 ± 0.29	0.56 ± 0.24^a^	0.54 ± 0.24^a^	0.53 ± 0.21^a^	0.60 ± 0.25^ad^	14.707	<0.001
VB (pmol/L)	331.71 ± 173.67	389.82 ± 154.43^a^	407.20 ± 163.28^a^	409.73 ± 168.56^a^	442.52 ± 227.81^ab^	6.507	<0.001
CYFRA 21-1 (ng/mL)	1.10 ± 0.51	1.11 ± 0.52	1.30 ± 0.81^ab^	1.54 ± 0.79^abc^	1.78 ± 0.86^abcd^	14.936	<0.001
SCC (ng/mL)	0.97 ± 0.38	0.96 ± 0.90	0.85 ± 0.40	0.87 ± 0.36	1.26 ± 0.51^abcd^	5.481	<0.001
Anti-TG (IU/mL)	1.46 ± 1.31	6.84 ± 31.02	5.98 ± 28.11	1.82 ± 3.11	2.21 ± 3.07	2.237	0.064
Anti-TPO (IU/mL)	0.54 ± 0.90	5.90 ± 59.90^a^	8.92 ± 65.25	2.19 ± 15.13^b^	0.97 ± 1.41	0.949	0.435
Ferritin (ng/mL)	137.79 ± 68.67	156.11 ± 74.25^a^	144.08 ± 74.23	143.06 ± 80.17	134.14 ± 91.88	1.458	0.214

Note: AP < 0.05 compared with the 18–24-year-old group; BP < 0.05 compared with the 25–39-year-old group; CP < 0.05 compared with the 40–49-year-old group; DP < 0.05 compared with the 50–64-year-old group.

RETRACTED

**Table 2:** A comparative study on the related parameters among different age groups of women in Qingdao, China ($\bar{x}$ ± *s*).

Groups	18–24 (*n* = 120)	25–39 (*n* = 120)	40–49 (*n* = 120)	50–64 (*n* = 120)	>65 (*n* = 60)	*F*	*P*
FBG (mmol/L)	4.66 ± 0.34	4.55 ± 0.38^a^	4.82 ± 0.41^ab^	5.05 ± 0.49^abc^	5.21 ± 0.44^abcd^	46.789	<0.001
ALT (IU/L)	12.01 ± 5.78	12.43 ± 5.84	16.63 ± 9.86^ab^	17.55 ± 7.56^ab^	16.65 ± 6.21^ab^	19.606	<0.001
AST (IU/L)	15.37 ± 3.67	14.66 ± 3.27	16.92 ± 5.13^ab^	18.64 ± 4.11^abc^	19.24 ± 4.34^abc^	28.114	<0.001
BUN (mmol/L)	4.27 ± 0.91	4.24 ± 1.01	4.83 ± 1.13^ab^	5.21 ± 1.17^abc^	5.64 ± 1.33^abcd^	31.985	<0.001
Cr (Umol/L)	83.46 ± 7.05	79.67 ± 8.50^a^	83.09 ± 8.10^b^	82.51 ± 7.19^b^	86.22 ± 7.93^bcd^	8.782	<0.001
Hb (g/L)	134.52 ± 8.54	132.621 ± 8.09	134.07 ± 9.84	137.32 ± 9.10^abc^	133.65 ± 8.27^d^	6.609	<0.001
TSH (uIU/mL)	2.04 ± 0.80	2.31 ± 1.09^a^	1.83 ± 0.85^ab^	2.04 ± 1.09^bc^	2.36 ± 1.37^c^	6.324	<0.001
FT3 (pmol/L)	4.45 ± 0.44	4.12 ± 0.51^a^	4.10 ± 0.63^a^	4.46 ± 0.39^bc^	4.35 ± 0.36^bc^	21.227	<0.001
TT3 (ng/mL)	1.09 ± 0.14	1.01 ± 0.17^a^	1.00 ± 0.17^a^	1.09 ± 0.12^bc^	1.09 ± 0.12^bc^	14.559	<0.001
FT4 (pmol/L)	13.82 ± 1.17	12.88 ± 1.36^a^	12.87 ± 1.49^a^	13.31 ± 1.08^abc^	13.22 ± 1.05^a^	15.963	<0.001
TT4 (*μ*g/dL)	8.22 ± 1.30	7.59 ± 1.16^a^	7.67 ± 1.21^a^	8.02 ± 1.06^bc^	7.87 ± 1.27	7.955	<0.001
VB12 (pmol/L)	412.56 ± 183.66	438.51 ± 178.20	507.16 ± 236.94^ab^	556.59 ± 245.61^abc^	480.22 ± 202.74^d^	11.874	<0.001
CYFRA 21-1 (ng/mL)	1.21 ± 0.63	1.36 ± 0.75	1.05 ± 0.56^b^	1.52 ± 1.86^ac^	1.55 ± 0.90^c^	4.509	0.001
SCC (ng/mL)	0.92 ± 0.34	0.95 ± 0.38	0.74 ± 0.28	1.00 ± 0.36	0.70 ± 0.30	0.563	0.690
Anti-TG (IU/mL)	12.05 ± 65.33	17.51 ± 67.93	19.04 ± 87.20	16.63 ± 73.09	2.16 ± 2.91	0.561	0.691
Anti-TPO (IU/mL)	5.97 ± 41.55	15.38 ± 80.93	30.20 ± 120.93^a^	10.06 ± 46.23^c^	0.35 ± 0.32^c^	2.796	0.025
Ferritin (ng/mL)	40.21 ± 33.81	46.82 ± 37.27	38.59 ± 30.89	77.62 ± 46.71^abc^	89.91 ± 60.37^abc^	37.155	<0.001

Note: AP < 0.05 compared with the 18–24-year-old group; BP < 0.05 compared with the 25–39-year-old group; CP < 0.05 compared with the 40–49-year-old group; DP < 0.05 compared with the 50–64-year-old group.

RETRACTED

**Table 3:** A comparative study of correlation parameters between males and females in the same age group of 18–24 years ($\bar{x}$ ± *s*).

Groups	Male (*n* = 120)	Female (*n* = 120)	*t*	*P*
FBG (mmol/L)	4.71 ± 0.35	4.66 ± 0.34	1.097	0.274
ALT (IU/L)	20.76 ± 12.63	12.01 ± 5.78	7.986	<0.001
AST (IU/L)	17.85 ± 4.88	15.37 ± 3.67	5.097	<0.001
BUN (mmol/L)	5.00 ± 0.97	4.27 ± 0.91	6.867	<0.001
Cr (Umol/L)	103.73 ± 7.82	83.46 ± 7.05	24.001	<0.001
Hb (g/L)	159.58 ± 8.28	134.52 ± 8.54	26.176	<0.001
TSH (uIU/mL)	1.89 ± 1.00	2.04 ± 0.80	−1.451	<0.001
FT3 (pmol/L)	4.99 ± 0.46	4.45 ± 0.44	10.452	<0.001
TT3 (ng/mL)	1.19 ± 0.14	1.09 ± 0.14	6.268	<0.001
FT4 (pmol/L)	14.35 ± 1.27	13.82 ± 1.17	3.795	<0.001
TT4 (*μ*g/dL)	8.20 ± 1.11	8.22 ± 1.30	−0.178	0.859
VB12 (pmol/L)	331.71 ± 173.67	412.56 ± 183.66	−26.309	<0.001
CYFRA 21-1 (ng/mL)	1.10 ± 0.51	1.21 ± 0.63	−1.658	0.098
SCC (ng/mL)	0.97 ± 0.38	0.92 ± 0.34	1.255	0.211
Anti-TG (IU/mL)	1.46 ± 1.31	12.05 ± 65.33	−1.958	0.051
Anti-TPO (IU/mL)	0.54 ± 0.90	5.97 ± 41.55	−1.549	0.122
Ferritin (ng/mL)	137.79 ± 68.67	40.21 ± 33.81	15.975	<0.001

**Table 4:** A comparative study of correlation parameters between male and female in the same age group of 25–39 years old ($\bar{x}$ ± *s*).

Groups	Male (*n* = 120)	Female (*n* = 120)	*t*	*P*
FBG (mmol/L)	4.66 ± 0.42	4.55 ± 0.38	2.489	0.013
ALT (IU/L)	23.56 ± 20.76	12.43 ± 5.84	11.057	<0.001
AST (IU/L)	19.03 ± 6.12	14.66 ± 3.27	8.172	<0.001
BUN (mmol/L)	5.15 ± 1.08	4.24 ± 1.01	7.885	<0.001
Cr (Umol/L)	101.35 ± 8.63	79.67 ± 8.50	22.768	<0.001
Hb (g/L)	155.60 ± 9.29	132.621 ± 8.09	23.830	<0.001
TSH (uIU/mL)	1.78 ± 0.81	2.31 ± 1.09	−4.974	<0.001
FT3 (pmol/L)	4.69 ± 0.44	4.12 ± 0.51	10.802	<0.001
TT3 (ng/mL)	1.12 ± 0.15	1.01 ± 0.17	5.974	<0.001
FT4 (pmol/L)	14.01 ± 1.27	12.88 ± 1.36	7.711	<0.001
TT4 (*μ*g/dL)	7.86 ± 1.24	7.59 ± 1.16	1.966	0.050
VB12 (pmol/L)	389.82 ± 154.43	438.51 ± 178.20	−28.965	<0.001
CYFRA 21-1 (ng/mL)	1.11 ± 0.52	1.36 ± 0.75	−3.161	0.002
SCC (ng/mL)	0.96 ± 0.90	0.95 ± 0.38	0.200	0.842
Anti-TG (IU/mL)	6.84 ± 31.02	17.51 ± 67.93	−1.751	0.081
Anti-TPO (IU/mL)	5.90 ± 59.90	15.38 ± 80.93	−1.160	0.247
Ferritin (ng/mL)	156.11 ± 74.25	46.82 ± 37.27	17.118	<0.001

**Table 5:** Comparison of correlation parameters between men and women of the same age group of 40–49 years old ($\bar{x}$ ± *s*).

Groups	Male (*n* = 120)	Female (*n* = 120)	*t*	*P*
FBG (mmol/L)	4.95 ± 0.46	4.82 ± 0.41	2.729	0.009
ALT (IU/L)	22.26 ± 20.76	16.63 ± 9.86	5.175	<0.001
AST (IU/L)	18.90 ± 5.35	16.92 ± 5.13	3.467	<0.001
BUN (mmol/L)	5.26 ± 1.09	4.83 ± 1.13	3.603	<0.001
Cr (Umol/L)	100.67 ± 10.06	83.09 ± 8.10	17.843	<0.001
Hb (g/L)	156.06 ± 8.27	134.07 ± 9.84	22.040	<0.001
TSH (uIU/mL)	1.79 ± 1.29	1.83 ± 0.85	−0.337	0.731
FT3 (pmol/L)	4.63 ± 0.41	4.10 ± 0.63	8.895	<0.001
TT3 (ng/mL)	1.09 ± 0.15	1.00 ± 0.17	4.991	<0.001
FT4 (pmol/L)	13.78 ± 1.15	12.87 ± 1.49	6.163	<0.001
TT4 (*μ*g/dL)	7.71 ± 1.25	7.67 ± 1.21	0.352	0.719
VB12 (pmol/L)	407.20 ± 163.28	507.16 ± 236.94	−23.765	<0.001
CYFRA 21-1 (ng/mL)	1.30 ± 0.81	1.05 ± 0.56	3.170	0.019
SCC (ng/mL)	0.85 ± 0.40	0.74 ± 0.28	2.942	0.466
Anti-TG (IU/mL)	5.98 ± 28.11	19.04 ± 87.20	−1.775	0.028
Anti-TPO (IU/mL)	8.92 ± 65.25	30.20 ± 120.93	−1.957	0.002
Ferritin (ng/mL)	144.08 ± 74.23	38.59 ± 30.89	17.672	<0.001

RETRACTED

**Table 6:** A comparative study of correlation parameters between males and females in the same age group of 50–64 years old ($\bar{x}$ ± *s*).

Groups	Male (*n* = 120)	Female (*n* = 120)	*t*	*P*
FBG (mmol/L)	5.18 ± 0.55	5.05 ± 0.49	2.262	0.010
ALT (IU/L)	21.24 ± 9.58	17.55 ± 7.56	3.872	<0.001
AST (IU/L)	19.26 ± 4.91	18.64 ± 4.11	1.226	0.252
BUN (mmol/L)	5.53 ± 1.22	5.21 ± 1.17	2.426	0.009
Cr (Umol/L)	101.24 ± 9.96	82.51 ± 7.19	19.646	<0.001
Hb (g/L)	154.92 ± 9.48	137.32 ± 9.10	17.008	<0.001
TSH (uIU/mL)	1.89 ± 1.22	2.04 ± 1.09	−1.185	0.731
FT3 (pmol/L)	4.70 ± 0.42	4.46 ± 0.39	5.316	<0.001
TT3 (ng/mL)	1.13 ± 0.16	1.09 ± 0.12	2.619	0.015
FT4 (pmol/L)	13.36 ± 1.24	13.31 ± 1.08	0.382	0.725
TT4 (*μ*g/dL)	7.84 ± 1.26	8.02 ± 1.06	−1.375	0.187
VB12 (pmol/L)	409.73 ± 168.56	556.59 ± 245.61	−24.834	<0.001
CYFRA 21-1 (ng/mL)	1.54 ± 0.79	1.52 ± 1.86	0.097	0.877
SCC (ng/mL)	0.87 ± 0.36	1.00 ± 0.36	−0.404	0.427
Anti-TG (IU/mL)	1.82 ± 3.11	16.63 ± 73.09	−2.428	0.016
Anti-TPO (IU/mL)	2.19 ± 15.13	10.06 ± 46.23	−1.963	0.274
Ferritin (ng/mL)	143.06 ± 80.17	77.62 ± 46.71	9.104	<0.001

**Table 7:** Correlation parameter comparison between males and females in the same age group of > 65 years old ($\bar{x}$ ± *s*).

Groups	Male (*n* = 60)	Female (*n* = 60)	*t*	*P*
FBG (mmol/L)	5.31 ± 0.78	5.21 ± 0.44	0.703	0.293
ALT (IU/L)	19.34 ± 11.24	16.65 ± 6.21	1.343	0.163
AST (IU/L)	20.95 ± 6.32	19.24 ± 4.34	1.457	0.085
BUN (mmol/L)	6.04 ± 1.55	5.64 ± 1.33	1.317	0.081
Cr (Umol/L)	100.88 ± 11.54	86.22 ± 7.93	6.841	<0.001
Hb (g/L)	150.08 ± 10.30	133.65 ± 8.27	8.275	<0.001
TSH (uIU/mL)	2.18 ± 1.26	2.36 ± 1.37	−0.678	0.402
FT3 (pmol/L)	4.40 ± 0.39	4.35 ± 0.36	0.659	0.592
TT3 (ng/mL)	1.07 ± 0.16	1.09 ± 0.12	−0.450	0.662
FT4 (pmol/L)	13.28 ± 1.13	13.22 ± 1.05	0.281	0.805
TT4 (*μ*g/dL)	7.59 ± 1.20	7.87 ± 1.27	−1.093	0.265
VB12 (pmol/L)	442.52 ± 227.81	480.22 ± 202.74	1.408	0.239
CYFRA 21-1 (ng/mL)	1.78 ± 0.86	1.55 ± 0.90	1.139	0.281
SCC (ng/mL)	1.26 ± 0.51	0.70 ± 0.30	5.350	0.086
Anti-TG (IU/mL)	2.21 ± 3.07	2.16 ± 2.91	0.074	0.997
Anti-TPO (IU/mL)	0.97 ± 1.41	0.35 ± 0.32	2.606	0.963
Ferritin (ng/mL)	134.14 ± 91.88	89.91 ± 60.37	2.617	<0.001

RETRACTED

**Table 8:** The reference range of male parameters in different age groups.

Groups		18–24 (*n* = 120)	25–39 (*n* = 120)	40–49 (*n* = 120)	50–64 (*n* = 120)	>65 (*n* = 60)
FBG (mmol/L)	P2.5	3.68	3.64	4.10	3.99	3.83
	P97.5	5.58	6.35	6.74	6.56	6.86

ALT (IU/L)	P2.5	6.00	5.00	4.00	8.00	5.00
	P97.5	64.00	65.00	61.00	68.00	69.00

AST (IU/L)	P2.5	9.00	10.00	11.00	3.00	8.00
	P97.5	36.00	44.00	50.00	37.00	49.00

BUN (mmol/L)	P2.5	3.00	2.00	3.25	3.04	2.25
	P97.5	8.59	8.15	9.30	10.69	10.73

Cr (Umol/L)	P2.5	85.00	76.00	68.80	66.90	83.00
	P97.5	124.00	121.00	126.00	129.00	135.00

Hb (g/L)	P2.5	141.00	134.00	131.00	132.00	129.00
	P97.5	189.00	181.00	176.00	184.00	173.00

TSH (uIU/mL)	P2.5	0.30	0.40	0.35	0.31	0.64
	P97.5	4.31	3.68	4.38	4.40	4.95

FT3 (pmol/L)	P2.5	4.09	3.69	3.70	3.81	3.64
	P97.5	6.36	5.79	5.67	5.86	5.23

TT3 (ng/mL)	P2.5	0.71	0.80	0.79	0.73	0.76
	P97.5	1.61	1.61	1.54	1.67	1.56

FT4 (pmol/L)	P2.5	11.15	11.09	10.65	11.08	10.69
	P97.5	18.08	17.97	17.52	17.12	15.66

TT4 (*μ*g/dL)	P2.5	5.33	4.25	5.31	4.88	5.03
	P97.5	11.52	10.77	11.58	11.27	11.52

VB12 (pmol/L)	P2.5	131.00	0.00	0.00	0.00	0.00
	P97.5	2.00	1.00	2.00	1.00	1.00

PROG (nmol/L)	P2.5	11.00	125.00	130.00	94.00	182.00
	P97.5	1383.00	947.00	1242.00	1107.00	1302.00

CYFRA 21-1 (ng/mL)	P2.5	0.26	0.35	0.32	0.39	0.75
	P97.5	3.07	3.29	5.96	4.76	4.74

SCC (ng/mL)	P2.5	0.40	0.20	0.30	0.30	0.70
	P97.5	2.60	9.90	3.10	2.50	2.90

Anti-TG (IU/mL)	P2.5	0.34	0.38	0.24	0.27	0.41
	P97.5	11.43	227.16	293.84	34.82	17.33

Anti-TPO (IU/mL)	P2.5	0.00	0.00	0.00	0.00	0.00
	P97.5	9.00	730.00	748.00	179.00	8.00

Ferritin (ng/mL)	P2.5	21.83	36.35	3.54	9.79	25.76
	P97.5	363.47	396.85	457.43	522.84	495.35

**Table 9:** Reference intervals of female parameters in different age groups.

Groups	RIs	18–24 (*n* = 120)	25–39 (*n* = 120)	40–49 (*n* = 120)	50–64 (*n* = 120)	>65 (*n* = 60)
FBG (mmol/L)	*P*_2.5_	3.93	3.83	3.99	4.31	4.32
	*P*_97.5_	5.23	5.37	5.65	6.19	6.13
ALT (IU/L)	*P*_2.5_	5.00	6.00	7.00	8.00	6.00
	*P*_97.5_	24.00	31.00	58.00	45.00	28.00
AST (IU/L)	*P*_2.5_	9.00	9.00	10.00	13.00	12.00
	*P*_97.5_	21.00	26.00	35.00	28.00	25.00
BUN (mmol/L)	*P*_2.5_	2.62	2.50	2.56	3.08	3.72
	*P*_97.5_	5.70	6.70	6.85	7.97	9.14
Cr (*μ*mol/L)	*P*_2.5_	71.00	65.00	66.00	69.00	74.00
	*P*_97.5_	98.00	94.00	102.00	99.00	102.00
Hb (g/L)	*P*_2.5_	119.0	115.0	116.0	120.0	115.0
	*P*_97.5_	148.0	148.0	155.0	155.0	150.0
TSH (*μ*IU/mL)	*P*_2.5_	0.66	0.82	0.65	0.58	0.61
	*P*_97.5_	3.54	5.59	4.13	4.92	5.91
FT3 (pmol/L)	*P*_2.5_	3.66	3.06	2.78	3.66	3.39
	*P*_97.5_	5.15	4.89	5.16	5.25	5.23
TT3 (ng/mL)	*P*_2.5_	0.86	0.74	0.69	0.86	0.87
	*P*_97.5_	1.34	1.27	1.37	1.31	1.37
FT4 (pmol/L)	*P*_2.5_	11.92	10.07	9.67	11.34	11.19
	*P*_97.5_	15.73	15.67	15.70	15.32	15.25
TT4 (*μ*g/dL)	*P*_2.5_	6.20	5.73	5.21	5.75	5.49
	*P*_97.5_	10.65	9.79	10.31	10.19	10.04
VB12 (pmol/L)	*P*_2.5_	165	176	179	202	244
	*P*_97.5_	773	809	926	987	989
CYFRA21-1 (ng/mL)	*P*_95_	3.16	2.80	2.04	2.76	3.74
SCC (ng/mL)	*P*_95_	1.99	1.50	1.30	1.28	1.20
Anti-Tg (IU/mL)	*P*_95_	2.43	2.39	2.41	2.45	2.50
Anti-TPO (IU/mL)	*P*_95_	0.82	0.72	0.75	0.76	0.70
Ferritin (ng/mL)	*P*_2.5_	4.70	4.78	3.10	6.15	21.29
	*P*_97.5_	98.00	135.50	140.50	200.11	225.00

RETRACTED

## Data Availability

The data used to support the findings of this study are included within the article.
